The article "Application of Pelvic Magnetic Resonance Imaging Scan Combined with Serum Pyruvate Kinase Isozyme M2, Neutrophil Gelatinase-Associated Lipocalin, and Soluble Leptin Receptor Detection in Diagnosing Endometrial Carcinoma" was published in 2022. Journal: Contrast Media Mol Imaging.

# Application of Pelvic Magnetic Resonance Imaging Scan Combined with Serum Pyruvate Kinase Isozyme M2, Neutrophil Gelatinase-Associated Lipocalin, and Soluble Leptin Receptor Detection in Diagnosing Endometrial Carcinoma

**DOI:** 10.1155/2022/7197505

**Published:** 2022-05-21

**Authors:** Shizhong Su, Liping Yin

**Affiliations:** ^1^Obstetrics and Gynecology, People's Liberation Army 960th Hospital, Jinan City 250000, Shandong Province, China; ^2^Imaging Department, Shandong Cancer Hospital and Institute, Shandong First Medical University and Shandong Academy of Medical Sciences, Jinan City 250117, Shandong Province, China

## Abstract

**Objective:**

To explore the application value of pelvic magnetic resonance imaging (MRI) scan combined with serum pyruvate kinase isozyme M2 (PKM2), neutrophil gelatinase-associated lipocalin (NGAL), and soluble leptin receptor (sOB-R) detection in diagnosing endometrial carcinoma (EC).

**Methods:**

The clinical data of 45 patients with pathologically confirmed EC treated in our hospital from May 2019 to May 2020 were retrospectively analyzed. All patients received pelvic MRI scan, serum PKM2, NGAL and sOB-R detection was performed, and the combination of the two was performed so as to analyze the diagnostic application value of the three modalities.

**Results:**

Compared with the joint detection, the number of true positive cases, sensitivity, specificity, and accuracy rate obtained by a single application of pelvic MRI or serum PKM2, NGAL, and sOB-R detection were obviously lower; the area under the ROC curve of the joint detection was obviously larger than that of single detection; the results of the joint detection were better than those of single detection (*P* < 0.05); the combined diagnosis obtained the highest sensitivity.

**Conclusion:**

Combining pelvic MRI with serum PKM2, NGAL, and sOB-4 detection can effectively promote the diagnostic accuracy for EC, presenting significant clinical diagnostic value.

## 1. Introduction

Endometrial carcinoma (EC) is an epithelial malignancy that occurs in the endometrium of women, which is classified into mucinous adenocarcinoma, endometrioid adenocarcinoma, papillary serous endometrial adenocarcinoma, adenocarcinoma with squamous cell differentiation, squamous carcinoma, and clear cell carcinoma [1, 2]. Relevant literature has pointed out that EC is one of the malignant tumors with high incidence worldwide, accounting for approximately 25% of malignant diseases of the female reproductive system [3]. Relevant data have revealed that EC, as a common pathological type, has a prevalence of 0.016%–0.019% [4]. In 2012, there were 319,588 new EC cases, ranking 6th in new cases of malignant tumors in women. Among them, 168,895 new EC cases were in European and American countries, ranking 4th, and 151,694 new EC cases were in developing countries, ranking 7th [5]. In the United States in 2015, there were 54,796 new EC cases and 10,109 cases died of EC, accounting for 55.79% of incidence and 33.38% of mortality among all gynecological cancers [6]. While in 2017, there were 61,379 new EC cases and 10,918 deaths from EC in the United States, the incidence was second only to colorectal cancer, lung cancer, and breast cancer, staying high in gynecological malignancies [7]. Recent studies have reported that the incidence of EC is increasing, and that its age of onset has been shown to be younger [8].

Although the incidence and mortality of EC are still high and the pathogenesis is still unclear, many scholars believe that EC is a gynecological tumor with a good prognosis [9]. EC is mainly characterized by abnormal vaginal bleeding and fluid drainage, and genetic factors, adverse lifestyles, and reproductive endocrine disorders are risk factors predisposing to the disease. Meanwhile, relevant literature has pointed out that currently about 69% of EC patients are diagnosed at an early stage of the disease, illustrating that the tumor is still located in the endometrium when diagnosed [10]. Such patients can achieve a 5-year overall survival rate of 93% after receiving clinical treatment [10]. Magnetic resonance imaging (MRI) has a high sensitivity in diagnosing EC, and its results have important implications in staging, providing guidance to clinical treatment [11]. However, MRI imaging is slower, requires more time and higher costs, and the diagnostic results of examination alone fail to meet clinical expectations. Also, some scholars believe that the detection of serum tumor markers in EC patients has similarly significant diagnostic value [12]. At present, clinical reports have confirmed the effectiveness of a single application of MRI as well as serum pyruvate kinase isozyme M2 (PKM2), neutrophil gelatinase-associated lipocalin (NGAL), and soluble leptin receptor (sOB-R) detection, while few reports focus on their combination. Based on this, the diagnosis modality combining MRI diagnosis with serum PKM2, NGAL, and sOB-R detection was adopted herein to provide more basis for future clinical treatment, with the results reported as follows.

## 2. Materials and Methods

### 2.1. General Data

The clinical data of 45 patients with pathologically confirmed EC treated in our hospital from May 2019 to May 2020 were retrospectively analyzed. The study met the World Medical Association Declaration of Helsinki [13].

### 2.2. Enrollment of Study Subjects

#### 2.2.1. Inclusion Criteria

(1) The patients were diagnosed with EC for the first time according to the comprehensive medical history, re-examination, ultrasound, and pathologic examination of endometrium, with the clinical manifestations of abnormal vaginal bleeding and fluid drainage; (2) the patients did not receive antitumor treatments such as radiotherapy and chemotherapy before surgery, did not use sexual hormones 180 d before visiting the hospital, and had complete hematological indexes; (3) the patients did not have signs of chronic/acute infections; (4) the patients did not have hematological diseases and autoimmune diseases; and (5) the patients did not have mental illness and could normally communicate with others.

#### 2.2.2. Exclusion Criteria

(1) The patients had endometriosis, endometrial polyp, and other benign lesions in the endometrium; (2) the patients had received dilatation and curettage; (3) the patients had incomplete clinical data and pathological examination results and were lost to postoperative follow-up; (4) the patients were complicated with tumor metastasis or other tumors; (5) the patients had pregnancy-related diseases and cervical diseases; (6) the patients were participating in other experiments.

### 2.3. Methods

#### 2.3.1. MRI Scan

The superconducting MRI scanner (manufacturer: Philips Medical Systems Nederland B.V.; model: Gyroscan Panorama) was used to perform examination on the patients. Before examination, the patients were advised repeatedly to fast for 4–6 h, properly fill the bladder, and remove all metal objects. Scanning sequences: (1) Axial, coronal and sagittal spin-echo (SE) T1WI (TR500 ms, TE8.1 ms); (2) axial and sagittal fast spin-echo (FSE) T2WI (TR4500 ms, TE81 ms), and coronal T2WI (TR4800 ms, TE120 ms), with a slice thickness of 3 mm, slice interval of 1 mm, and the number of signal-averaged = 1; (3) DWI (TR3500, TE75 ms), the dispersed factor *b* values were 0 s/mm^2^ and 1,000 s/mm^2^, with slice interval of 1 mm, a slick thickness of 3 mm, FOV of 22 cm ∗ 22 cm, and a number of signal-averaged = 10; (4) a three-dimensional volumetric interpolated fast spoiled GRE T1WI (VIBE) sequence for DCE-MR, and the appropriate slice on the sagittal T2WI was selected, with TR4.05 ms, TE1.85 ms, slice thickness of 3 mm, FOV of 35 cm ∗ 35 cm, number of signal-averaged = 1, and total 20 time phases. The nonintermittent scanning was performed, with 10 s for each time phase. Gd-DTPA (0.1 mmol/kg) was injected through the cubital vein using a dual-barrel dual-channel special high-pressure injector for MR at a flow rate of 2 ml/s. Dynamic contrast-enhanced time-phase scans were initiated before drug injection, and the injection was finished after the end of the first time-phase scan. After dynamic contrast-enhanced scans, transaxial, sagittal, and coronal postenhancement scans were performed using a fat-suppressed sequence.

#### 2.3.2. Serum PKM2, NGAL, and sOB-R Detection

Five ml of fasting venous blood was drawn from all patients and preserved in EDTA anticoagulation test tubes for 10-min centrifugation at 3,000 r/min and then let stand for 20 min, after that, the upper serum was separated and stored in the −80°C freezer and then sent for detection within 1 h. The patients' serum PKM2, NGAL, and sOB-R indicators were detected by the enzyme-linked immunosorbent assay (ELISA), the standard detection was carried out in strict accordance with the specification and instructions on the kits (manufacturer: MSK Biology Company).

### 2.4. Observation Indexes

The numbers of true-positive cases, false-positive cases, true-negative cases, and false-negative cases obtained by a single application of pelvic MRI scan, serum PKM2, NGAL, and sOB-R detection, and their combination were compared.

The sensitivity, specificity, and accuracy of single application of pelvic MRI scan, serum PKM2, NGAL, and sOB-R detection, and their combination were compared. Sensitivity = number of true-positive cases/(number of true-positive cases + number of false-negative cases) ∗  100%, specificity = number of true-negative cases/(number of true-negative cases + number of false-positive cases) ∗ 100%, and accuracy = number of accurately diagnosed cases/total number of cases ∗ 100%.

The utility of the three diagnosis modalities was compared by plotting the ROC curve.

### 2.5. Statistical Processing

In this study, the statistical analysis and processing of experimental data were conducted by the software SPSS21.0, the picture drawing software was GraphPad Prism 7 (GraphPad Software, San Diego, USA), the enumeration data were examined by *X*^2^ test and expressed by (*n* (%)), the measurement data were examined by *t*-test and expressed by ($\bar{x}\pm s$), and differences were considered statistically significant at *P* < 0.05.

## 3. Results

### 3.1. Statistics of Baseline Data of All Subjects

Table 1 showed the statistics of baseline data of all subjects.

### 3.2. Comparison of Numbers of True-Positive Cases, False-Positive Cases, True-Negative Cases, and False-Negative Cases between Single Detection and Combined Detection

Table 2 showed that the numbers of true-positive cases of pelvic MRI scan and single detection of serum PKM2, NGAL, and sOB-R were obviously lower than that of combined detection.

### 3.3. Comparison of Sensitivity and Specificity between Single Detection and Combined Detection

Table 3 showed that the sensitivity, specificity, and accuracy rate of single detection were obviously lower than those of combined detection.

### 3.4. Area under ROC Curve of Single Detection and Combined Detection

Figure 1 showed that the area under the ROC curve of combined detection was obviously larger than that of single detection.

### 3.5. Comparison of Areas, S.E.^a^, Asymp. Sig.^b^, and Asymp. 95% CI of Various Indicators

The results of joint detection were better than those of single detection (*P* < 0.05) (see Table 4.

### 3.6. Comparison of Sensitivity and 1-Specificity

Table 5 showed that the joint detection obtained the highest sensitivity.

## 4. Discussion

Relevant literature has pointed out that the incidence of EC varies in different regions and countries, which is significantly higher in developed countries such as Europe and the United States than in developing countries, and accounts for approximately 49% of gynecological malignancies [14]. Fu et al. [15] stated that in China, the incidence of EC was significantly higher in more developed cities such as Shanghai and Beijing. Some published works demonstrated that in 2015, EC has become the malignant tumor with the highest incidence among the female reproductive system diseases in Beijing, ranking 5th in the female malignant tumors in Beijing, and its incidence shows an increasing trend (16.18/100,000 to 17.52/100,000) [16]. Antonio et al. [17] stated that the 5-year survival rates of EC patients at stage I, II, III, and IV were, respectively, 95.79%, 94.69%, 71.29%, and 23.79%, and considered that the survival rate of EC was significantly associated with pathological type, histological grade, and presence or absence of lymphatic metastasis. Meanwhile, Varol et al. [18] pointed out that the prognosis of EC disease is related to the degree of differentiation, clinical stages, and presence or absence of metastasis, and that the main cause of death of this disease is blood and lymph metastasis causing dysfunction in other organs. At present, the clinical treatment of the disease mainly focuses on “early diagnosis and early treatment,” the prognosis of EC can be greatly improved if EC patients are diagnosed at an early stage due to clinical manifestations such as abnormal vaginal bleeding, and endometrial sampling followed by the pathological diagnosis is the most accurate way for EC diagnosis [19]. In recent years, MRI, as the optimal preoperative imaging examination, is widely used in clinical diagnosis. MRI exhibits high sensitivity in diagnosing EC and can provide effective staging data for clinical treatment, thereby providing correct guidance. In addition, the utility of MRI diagnosis has been confirmed in nasopharyngeal carcinoma, prostate cancer, breast cancer, and cervical cancer [20]. Endometrial tumors can be revealed by MRI imaging, by adjusting the imaging parameters, the tissue contrast can be effectively enhanced and the depth of tumor invasion into the uterine stroma can be better evaluated, and in this process, MRI can reveal the corresponding area by locating the required imaging plane, and at the same time, through enhanced T1WI, T2WI and dynamic contrast-enhanced MRI, patients' tumors and lesions can be determined. Therefore, MRI has a positive role in identifying EC [21]. Some studies have confirmed that MRI has a high diagnostic value in detecting adenomyosis and endometrial hyperplasia diseases [22]. Meanwhile, some scholars also believe that the detection of serum indicators in EC patients is also beneficial to the analysis of patient condition, and the reason is that PKM2 is a phosphorylase, which can phosphorylate more than 100 proteins in the human body, and it is also a marker of tumor energy metabolism conversion, presenting up-regulated expression in most cancers [23]. NGAL is a new member of the lipocalin family in human body. Its high expression is closely related to the migration, proliferation and invasion of malignant cells, so it is often used to aid the diagnosis of malignant tumors. High expression of sOB-R is associated with the occurrence and progression of EC, and all EC cell lines express higher levels of sOB-R. Although single application of MRI scan or serum detection presents higher diagnostic value, erroneous diagnosis or missed diagnosis may still occur in some patients.

With the advancement of medical technology, some scholars have pointed out that combining MRI scan with serum detection can obtain better results than single detection [24, 25]. In this study, the numbers of true positive cases detected by single detection of pelvic MRI scan and serum PKM2, NGAL, and sOB-R were obviously lower than that of joint detection, and the sensitivity, specificity and accuracy rate were also obviously lower in single detection than in joint detection, indicating that applying the diagnostic modalities such as pelvic MRI scan and serum PKM2, NGAL and sOB-R detection alone did not obtain desirable diagnostic efficacy and high diagnostic sensitivity, specificity and accuracy rate, and that the joint detection achieved better diagnostic results because it could provide more rich positive diagnostic information in clinic through different means. In addition, as many factors such as bacterial infection and other inflammations can affect serum indicators, the detection of serum PKM2, NGAL and sOB-R alone cannot accurately determine EC and needs to be used in combination with pelvic MRI scan to complement each other and improve the diagnostic performance. The study results also showed that compared with single detection, the joint detection had obviously larger area under ROC curve, better results (*P* < 0.05), and the highest sensitivity, which fully demonstrated that the joint detection has a higher accuracy rate and further improves the clinical diagnostic value. Shortcomings of the study: First, there was selection bias inherent to retrospective study, such as differences in staff technique for performing MRI examination and preoperative histopathologic examination; second, this trial did not include patients who received conservative treatment and nonsurgical treatment, and did not consider the prognosis of the patients; and finally, this study was based on the population within the region and did not include sufficient amount of patients from other provinces, so the results might be affected by the small sample size and regional culture. Therefore, it is necessary to further improve the study protocol, increase the sample size, and develop multicenter studies. In the near future, with the continuous improvement and advancement of medical technology, a technique for the effective diagnosis of EC disease may be explored to provide more evidence-based basis for the clinical treatment of such patients.

## Figures and Tables

**Figure 1:** Area under ROC curve of single detection and combined detection.

**Table 1:** Statistics of baseline data of all subjects.

Item	Number of cases	Proportion (%)
Mean age ($\bar{x}\pm s$, years)	53.59 ± 10.40	—
BMI ($\bar{x}\pm s$, kg/m^2^)	20.56 ± 0.84	—
Course of disease (months)	11.86 ± 6.17	—
Menopause		
Yes	30	66.67
No	15	33.33
FIGO stage (number of cases)		
Stage (0) carcinoma in situ	8	17.78
Stage I	11	24.44
Stage II	13	28.89
Stage III	7	15.56
Stage IV	6	13.33
Degree of tumor differentiation		
Poor	18	40.00
Moderate	17	37.78
Well	10	22.22
Complicated with lymphatic metastasis		
Yes	36	80.00
No	9	20.00
Occupation		
Teacher	11	24.44
Civil servant	10	22.22
Accountant	13	28.89
Self-employed	8	17.78
Others	3	6.67
Family economic status		
≥3,000 yuan/(month·person)	30	66.67
<3,000yuan/(month·person)	15	33.33
Place of residence		
Urban area	25	55.56
Rural area	20	44.44
Educational degree		
College	30	66.67
Middle school	10	22.22
Primary school	5	11.11
Nationality		
Han	40	88.89
Others	5	11.11

**Table 2:** Comparison of numbers of true-positive cases, false-positive cases, true-negative cases, and false-negative cases between single detection and combined detection (*n* (%)).

Detection modality	True positive (cases)	False positive (cases)	True negative (cases)	False negative (cases)
Pelvic MRI scan	33 (73.33%)^*∗*^	4 (8.89%)	5 (11.11%)	3 (6.67%)
Serum PKM2, NGAL, and sOB-R	27 (60.00%)^#^	6 (13.33%)	5 (11.11%)	7 (15.56%)^##^
Combined detection	41 (91.11%)	1 (2.22%)	2 (4.44%)	1 (2.22%)

^*∗*^Obvious difference in numbers of true-positive cases between pelvic MRI scan and combined detection (*x*^2^ = 4.865, *P* < 0.05); ^#^Obvious difference in numbers of true-positive cases between serum PKM2, NGAL, and sOB-R detection and combined detection (*x*^2^ = 11.791, *P* < 0.05); and ^##^Obvious difference in numbers of false-positive cases between serum PKM2, NGAL, and sOB-R detection and combined detection (*x*^2^ = 4.939, *P* < 0.05).

**Table 3:** Comparison of sensitivity, specificity, and accuracy rate between single detection and combined detection (*n* (%)).

Detection modality	Sensitivity (%)	Specificity (%)	Accuracy rate (%)
Pelvic MRI scan	91.67	55.56	33 (73.33%)
Serum PKM2, NGAL, and sOB-R detection	79.41	45.45	27 (60.00%)
Combined detection	97.62	66.67	41 (91.11%)

**Table 4:** Comparison of areas, S.E.^a^, Asymp. Sig.^b^, and Asymp. 95% CI of various indicators.

				Asymp. 95% CI	
Test result variables	Area	S.E.^a^	Asymp. Sig.^b^	Lower limit	Upper limit
Pelvic MRI scan	0.753	0.075	0.004	0.605	0.901
Serum PKM2, NGAL, and sOB-R	0.619	0.085	0.172	0.453	0.785
Joint detection	0.887	0.056	<0.001	0.778	0.996

**Table 5:** Comparison of sensitivity and 1-specificity.

Test result variables	Positive^a^ if greater than or equal to	Sensitivity	1-specificity
Pelvic MRI scan	−1.0000	1.000	1.000
	0.5000	0.714	0.208
	2.0000	<0.001	<0.001

Serum PKM2, NGAL, and sOB-R detection	−1.0000	1.000	1.000
	0.5000	0.571	0.333
	2.0000	<0.001	<0.001

Joint detection	−1.0000	1.000	1.000
	0.5000	0.857	0.083
	2.0000	<0.001	<0.001

## Data Availability

The data to support the findings of this study are available on reasonable request from the corresponding author.

## References

[1] Buchynska L. G., Borykun T. V., Iurchenko N. P., Nespryadko S. V., Nesina I. P. (2020). Expression of microRNA in tumor cells of endmetrioid carcinoma of endometrium. *Experimental Oncology*.

[2] Norimatsu Y., Irino S., Maeda Y. (2021). Nuclear morphometry as an adjunct to cytopathologic examination of endometrial brushings on LBC samples: a prospective approach to combined evaluation in endometrial neoplasms and look alikes. *Cytopathology*.

[3] Euscher E. D., Duose D. Y, Lan C (2020). Mesonephric-like carcinoma of the endometrium. *The American Journal of Surgical Pathology*.

[4] Kaur R., Mehta J., Borges A. M. (2021). Role of SMARCA4 (BRG1) and SMARCB1 (INI1) in dedifferentiated endometrial carcinoma with paradoxical aberrant expression of mmr in the well-differentiated component: a case report and review of the literature. *International Journal of Surgical Pathology*.

[5] Sangwan K., Garg M., Pathak N., Bharti L. (2020). Expression of cyclin D1 in hyperplasia and carcinoma of endometrium and its correlation with histologic grade, tumor type, and clinicopathological features. *Journal of Laboratory Physicians*.

[6] Iida T., Muramatsu T., Kajiwara H. (2020). Small cell neuroendocrine carcinoma of the endometrium with difficulty identifying the original site in the uterus. *Tokai Journal of Experimental & Clinical Medicine*.

[7] Wong R. W. C., Talia K. L., McCluggage W. G. (2020). Endometrial gastric-type carcinoma. *The American Journal of Surgical Pathology*.

[8] Liu Y., Chang Y., Cai Y.-x (2020). Inhibition of lnc-OC1 induced cell apoptosis and decreased cell viability by releasing miR-34a and inhibiting PD-L1 in endometrial carcinoma. *Reproductive Sciences*.

[9] Badary D. M., Abou-Taleb H. (2020). Vitamin D receptor and cellular retinol-binding protein-1 immunohistochemical expression in normal, hyperplastic and neoplastic endometrium: possible diagnostic and therapeutic implications. *Annals of Diagnostic Pathology*.

[10] Tasuku M., Kubo T., Yoshihiko H. (2021). Less correlation between mismatch repair proteins deficiency and decreased expression of HLA class I molecules in endometrial carcinoma: a different propensity from colorectal cancer. *Medical Molecular Morphology*.

[11] Kazuhiro K., Takako K., Kawanaka Y (2021). Characteristics of MR imaging for staging and survival analysis of neuroendocrine carcinoma of the endometrium: a multicenter study in Japan. *Magnetic Resonance in Medical Sciences*.

[12] O’Toole S. A., Huang Y., Norris L. (2021). HE4 and CA125 as preoperative risk stratifiers for lymph node metastasis in endometrioid carcinoma of the endometrium: a retrospective study in a cohort with histological proof of lymph node status. *Gynecologic Oncology*.

[13] World Medical Association (2013 Nov 27). World medical association declaration of Helsinki. *JAMA*.

[14] Travaglino A., Raffone A., Gencarelli A. (2021). Clinico-pathological features associated with mismatch repair deficiency in endometrial undifferentiated/dedifferentiated carcinoma: a systematic review and meta-analysis. *Gynecologic Oncology*.

[15] Fu D.-J., De Micheli A. J., Bidarimath M. (2020). Cells expressing PAX8 are the main source of homeostatic regeneration of adult endometrial epithelium and give rise to serous endometrial carcinoma. *Disease models & mechanisms*.

[16] Xu S., Yang Y., Wang X. (2020). *γ*-Glutamyl cyclotransferase contributes to endometrial carcinoma malignant progression and upregulation of PD-L1 expression during activation of epithelial-mesenchymal transition. *International Immunopharmacology*.

[17] Antonio T., Antonio R., Annarita G., Antonio M., Fulvio Z., Luigi I. (2020). Endometrial gastric-type carcinoma: an aggressive and morphologically heterogenous new histotype Arising from gastric metaplasia of the endometrium. *The American Journal of Surgical Pathology*.

[18] Varol G., Mustafa K., İsa Aykut Ö., Ilker C., Muzaffer S., Kemal G. (2020). Do estrogen, progesterone, P53 and Ki67 receptor ratios determined from curettage materials in endometrioid-type endometrial carcinoma predict lymph node metastasis. *Current Problems in Cancer*.

[19] Christine S., Oluwole F. (2020). High-grade endometrioid carcinoma of the endometrium with a GATA-3-positive/PAX8-negative immunophenotype metastatic to the breast: a potential diagnostic pitfall. *International Journal of Surgical Pathology*.

[20] Xu Z., Tian Y., Fu J., Xu J., Bao D., Wang G. (2020). Efficacy and prognosis of fertility-preserved hysteroscopic surgery combined with progesterone in the treatment of complex endometrial hyperplasia and early endometrial carcinoma. *Journal of B.U.ON.: Official Journal of the Balkan Union of Oncology*.

[21] Cuevas D., Velasco A., Vaquero M. (2020). Intratumour heterogeneity in endometrial serous carcinoma assessed by targeted sequencing and multiplex ligation-dependent probe amplification: a descriptive study. *Histopathology*.

[22] Rivera G., Niu S., Chen H., Fahim D., Peng Y. (2020). Collision tumor of endometrial large cell neuroendocrine carcinoma and low-grade endometrial stromal sarcoma: a case report and review of the literature. *International Journal of Surgical Pathology*.

[23] Vroobel K. M., Attygalle A. D. (2020). Sarcomatous transformation in undifferentiated/dedifferentiated endometrial carcinoma: an underrecognized phenomenon and diagnostic pitfall. *International Journal of Gynecological Pathology*.

[24] Dai Y., Chen W., Xu X. (2022). Factors affecting adenoma risk level in patients with intestinal polyp and association analysis. *Journal of Healthcare Engineering*.

[25] Zhang C., Shao S., Zhang Y. (2020). LncRNA PCAT1 promotes metastasis of endometrial carcinoma through epigenetical downregulation of E-cadherin associated with methyltransferase EZH2. *Life Sciences*.

